The article "Long non-coding RNA nuclear enriched abundant transcript 1 (NEAT1) sponges microRNA-124-3p to up-regulate phosphodiesterase 4B (PDE4B) to accelerate the progression of Parkinson’s disease" was published in 2021. Journal: Bioengineered.

# Long non-coding RNA nuclear enriched abundant transcript 1 (NEAT1) sponges microRNA-124-3p to up-regulate phosphodiesterase 4B (PDE4B) to accelerate the progression of Parkinson’s disease

**DOI:** 10.1080/21655979.2021.1883279

**Published:** 2021-02-22

**Authors:** Ming-Yu Chen, Kai Fan, Lian-Jiang Zhao, Jie-Mei Wei, Ji-Xu Gao, Zhen-Fu Li

**Affiliations:** a Department of Neurology, Linyi Central Hospital, Linyi City Shandong, China; b Department of Neurology, The Third People’s Hospital of Linyi, Linyi City Shandong, China; c Department of Laboratory, Linyi Cancer Hospital, Linyi City Shandong, China

**Keywords:** PD, neat1, miR-124-3p, pde4b

## Abstract

Reportedly, long non-coding RNA (lncRNA) are crucial modulators in neurodegenerative diseases. Herein, we investigated the role of lncRNA nuclear enriched abundant transcript 1 (NEAT1) in Parkinson’s disease (PD). *In-vitro* PD model was established based on SH-SY5Y cells treated with 1-methyl-4-phenylpyridinium (MPP+). NEAT1, microRNA (miR) −124-3p and phosphodiesterase 4B (PDE4B) expression levels were examined by qRT-PCR. CCK-8 assay and LDH release assay were adopted to delve into the cell viability and cytotoxicity, respectively. Besides, western blot was utilized to determine mTOR, p-mTOR and PDE4B expression levels. ELISA was executed to detect the levels of tumor necrosis factor α (TNF-α), interleukin 1β (IL-1β) and interleukin 6 (IL-6). Dual-luciferase reporter assay and RIP assay were used to probe the relationship between miR-124-3p and NEAT1 or PDE4B. We demonstrated that, in SH-SY5Y cells treated with MPP+, NEAT1 and PDE4B expression levels were raised, while miR-124-3p expression was repressed; NEAT1 depletion or miR-124-3p overexpression increased the cell viability and suppressed cell injury. Besides, miR-124-3p was confirmed as the direct target of NEAT1, and its down-regulation counteracted the impact of NEAT1 depletion on SH-SY5Y cells. PDE4B was as the downstream target of miR-124-3p, and its overexpression weakens the impact of miR-124-3p on SH-SY5Y cells. Additionally, NEAT1 decoyed miR-124-3p to modulate PDE4B expression. Collectively, in MPP+-induced SH-SY5Y cells, NEAT1 depletion increases cell viability, represses cytotoxicity and reduces inflammatory response by regulating miR-124-3p and PDE4B expression levels, suggesting that NEAT1 may be a promising target for treating PD.

## Introduction

Parkinson’s disease (PD) is a prevailing neurodegenerative disorder [1]. Its pathological features are the loss of dopaminergic (DA) neurons in substantia nigra pars compacta (SNpc), and the extensive accumulation of intracellular α-Synuclein (α-SYN), leading to motor coordination disorders and cognitive impairment [2]. It is reported that the decrease of mitochondrial function, imbalance of α-synuclein protein homeostasis, excessive production of oxidative stress, imbalance of calcium homeostasis, activation of apoptosis cascade, and neuroinflammation are implicated in the pathogenesis of PD [3]. Drug treatment and deep brain stimulation techniques can improve the life quality of the patients [4]. However, the detailed molecular mechanism of PD pathogenesis is still obscure.

Long non-coding RNAs (lncRNAs) are transcripts with exceeding 200*nt* which cannot encode proteins. LncRNAs are participants in diverse biological processes via various mechanisms [5,6]. Recently, some lncRNAs have been considered as therapy targets for neurodegenerative diseases, like PD [7,8]. For instance, lncRNA AL049437 knockdown can reduce 1-methyl-4-phenylpyridinium (MPP+)-induced neuronal injury in SH-SY5Y cells via modulating miR-205-5p/MAPK1 axis [9]. LncRNA SNHG1 aggravates MPP+-induced cytotoxicity of SH-SY5Y cells via modulating miR-153-3p/PTEN/AKT/mTOR axis [10]. Reportedly, lncRNA nuclear enriched abundant transcript 1 (NEAT1) aggravates Aβ-induced neuronal injury in Alzheimer’s Disease [11]. Interestingly, NEAT1 expression is elevated in 1-Methyl-4-phenyl-2, 3, 6-tetrahydropyridine (MPTP)-induced PD mice, and its knockdown can reduce the ratio of Bax to Bcl-2, the activity of caspase-3 and α-synuclein expression in neurons to exert ameliorative effects [12]. *In vitro*, NEAT1 depletion can inhibit the expression and release of IL-1β, IL-6 and TNF- α, suppress the neuronal apoptosis and increase neuronal viability [13]. However, the molecular mechanism by which NEAT1 participates in PD progression is still inconclusive.

MicroRNAs (miRNAs) are known as endogenous single-stranded non-coding transcripts with about 22*nt*, which can regulate downstream genes’ expression by binding with the 3ʹUTR of mRNA [14]. MiRNAs play certain roles in diverse diseases, including neurodegenerative diseases [15,16]. For example, reportedly, crocin exhibits neuroprotective impacts in rotenone-induced PD in rats via activating PI3K/Akt/mTOR axis and enhancing the expression levels of miR-7 and miR-221 [17]. MiR-425 defect contributes to necroptosis of dopaminergic neurons [18]. MiR-124 modulates cell survival, apoptosis, autophagy, oxidative damage, mitochondrial dysfunction and neuroinflammation through various pathways, and it is considered as a potential therapy target for PD [19].

Here, we adopted MPP+ to treat SH-SY5Y cells to establish an *in-vitro* PD model. This work was designed to confirm the impact of NEAT1 on the growth and apoptosis of neurons, and delve into the molecular regulatory mechanism of NEAT1, which is helpful to further understand the pathogenesis of PD and pave way for its clinical diagnosis and treatment.

## Materials and methods

### Cell culture and treatments

The America Type Culture College (ATCC, Manassas, VA, USA) was the supplier of human neuroblastoma cell line SH-SY5Y and embryonic kidney epithelial cell line HEK-293 T, both of which were cultured in Dulbecco’s Modified Eagle Medium (Invitrogen, Carlsbad, CA, USA) containing with 10% fetal bovine serum (Invitrogen), 100 U/mL penicillin and 100 μg/mL streptomycin (Invitrogen). To establish *in-vitro* PD model, SH-SY5Y cells were subsequently treated with diverse concentrations (0, 250, 500, 1000 or 2000 μM) of MPP+ (Sigma-Aldrich, Beijing, China) for 48 h, or 1000 μM of MMP+ for different times (0, 12, 24, 48 or 72 h).

### Cell culture and transfection

Small interfering RNA (siRNA) against NEAT1 (si-NEAT1), siRNA against PDE4B (si-PDE4B), siRNA negative control (si-NC), NEAT1 overexpression vector, PDE4B overexpression vector, pcDNA empty vector (pcDNA), miR-124-3p mimic, mimic negative control (miR-NC), miR-124-3p inhibitor, and inhibitor control (NC inhibitor) (sequences are detailed in Table 1) were available from GenePharma (Shanghai, China). Cell transfection was carried out with Lipofectamine™ 2000 transfection reagent (Invitrogen) 48 h before MPP+ treatment.

**Table 1.** The sequences of the miRNAs used in this study

Targets	Sequence
**miR-124-3p mimic**	5ʹ-UAAGGCACGCGGUGAAUGCCCA-3’
**mimic negative control (miR-NC)**	5ʹ-UUCUCCGAACGUGUCACGUTT-3ʹ
**miR-124-3p inhibitor**	5ʹ-GGCAUUCACCGCGUGCCUUA-3’
**inhibitor negative control (anti-miR-NC)**	5ʹ-CAGUACUUUUGUGUAGUACA-3ʹ

### Quantitative real-time polymerase chain reaction (qRT-PCR)

Total RNA was isolated with TRIzol reagent (Invitrogen) from SH-SY5Y cells. With total RNA as template, cDNA was subsequently synthesized with One Step PrimeScript cDNA synthesis kit (Takara, Dalian, China). Next, qRT-PCR was performed by SYBR® Premix Ex TaqTM II (Takara) on an ABI 7500 real-time PCR system (Applied Biosystems, Foster City, CA, USA), with β-actin as the internal control for NEAT1 and PDE4B mRNA, and U6 as that for miR-124-3p. The sequences are detailed in Table 2.

**Table 2.** The sequences of the primers used in this study

Primers	Forward	Reverse
**NEAT1**	5ʹ-TGGCTAGCTCAGGGCTTCAG-3ʹ	5ʹ-TCTCCTT GCCAAGCTTCCTTC-3ʹ
**PDE4B**	5ʹ- CTATACCGATCGCATTCAGGTC-3ʹ	5ʹ- CTGTCCATTGCCGATACAATT-3ʹ
**β-actin**	5ʹ-TGAGCGCGGCTACAGCTT-3’	5ʹ-TCCTTAATGTCACGCACGATTT-3’
**miR-124-3p**	5ʹ-TCTTTAAGGCACGCGGTG-3’	5ʹ-TATGGTTTTGACGACTGTGTGAT-3’
**U6**	5ʹ-TGCTTCGGCAGCACATATAC-3’	5ʹ-ATGGAACGCTTCACGAATTT-3’

### Cell viability assay

The viability of SH-SY5Y cells was examined by MTT assay. In short, 2 × 10^3^ SH-SY5Y cells were inoculated into each well of a 96-well plate with 0.5 mg/ml MTT solution (Sigma-Aldrich, Beijing, China), and following that, the cells were incubated at 37°C in 5% CO_2_ for 4 h. Next, the supernatant was immediately removed, with 150 μl of dimethyl sulfoxide (DMSO) (Sigma-Aldrich, Beijing, China) loaded into each well. Then, the formazan was dissolved after shaking, and the OD_490nm_ of the wells was measured by a microplate reader (Bio-Rad, Hercules, CA, USA).

### Lactate dehydrogenase (LDH) assay

The LDH release was detected by a microplate reader using LDH-cytotoxicity assay kit (Abcam Shanghai, China) to evaluate the injury of the cells according to the manufacturer’s instruction.

### Enzyme-linked immunosorbent assay (ELISA)

To probe the release of inflammatory cytokines, tumor necrosis factor α (TNF-α), interleukin 1β (IL-1β), and interleukin 6 (IL-6) levels in the supernatant of SH-SY5Y cells were determined by ELISA kits (Beyotime, Shanghai, China) according to the protocol, respectively.

### Western blot

10 μg of total protein extracted by RIPA lysis buffer (Beyotime, Shanghai, China) in each group was subjected to SDS-PAGE and subsequently transferred to polyvinylidinefluoride membrane (Millipore, Billerica, MA, USA), which was then blocked by 5% skimmed milk and incubated with the primary antibodies [anti-p-mTOR (1: 500, ab109268, Abcam), anti-mTOR (1: 1000, ab2732, Abcam), anti-PDE4B (1:1000, ab14611, Abcam) and anti-GAPDH (1:1000, ab8245, Abcam)] at 4°C overnight. Next, the membrane was incubated with the corresponding secondary antibodies (Beyotime, Shanghai, China) for 1 h at room temperature. After the membranes were washed in 1× TBST, the protein bands were developed with enhanced chemiluminescent substrate (Thermo Scientific, Carlsbad, CA, USA), and ultimately, the gray value was analyzed by Image J software (NIH-Image, Bethesda, MD, USA).

### Dual-luciferase activity assay

Wild-type (WT) or mutant (MUT) NEAT1 fragment with miR-124-3p binding site and the WT or MUT 3ʹUTR of PDE4B with the putative binding site of miR-124-3p were respectively amplified through PCR and accordingly inserted into the downstream region of luciferase reporter vector pGL3 (Promega, Madison, WI, USA) to establish recombinant luciferase reporters. Next, the luciferase reporters (NEAT1-WT, NEAT1-MUT, PDE4B-WT and PDE4B-MUT) were, respectively, transfected into HEK-293 T cells with miR-NC or miR-124-3p. 48 h later, firefly luciferase activity was standardized to renilla luciferase activity with the luciferase reporter assay system (Promega, Madison, WI, USA).

### RIP assay

RIP assay was operated by EZ Magna RIP kit (Millipore, Bedford, MA, USA). Generally, 100 μl of RIP lysis buffer containing 0.25 μl RNase and 0.5 μl protease inhibitor was adopted to lyse SH-SY5Y cells. Then, the cell lysates were incubated with anti-Argonaute 2 (Ago2) or IgG antibody coupled magnetic beads (Millipore, Bedford, MA, USA). After that, the mixture was incubated with proteinase K. Subsequently, the RNA, with TRIzol method, was extracted from the immunoprecipitate, and NEAT1 and miR-124-3p expression levels were probed by qRT-PCR.

### RNA pull-down assay

According to the manufacturer’s instruction, biotin-labeled NEAT1 (Bio-NEAT1) or Bio-NC (Millipore, Bedford, MA, USA) was respectively transfected into cells. 48 h later, the cell lysate was incubated with streptavidin agarose-magnetic beads at 4°C for 1 h. Ultimately, the miR-124-3p content in bead-RNA complex was probed by qRT-PCR.

### Statistical analysis

All of the data were generally expressed as ‘mean ± standard deviation’ and statistically processed by SPSS 17.0 software (SPSS Inc., Chicago, IL, USA) and Graph Prism 5.0 software (GraphPad Prism, San Diego, California). Student’s *t* test and one-way ANOVA were adopted for comparing the data. Statistically, *P* < 0.05 was meaningful.

## Results

### NEAT1 is raised and miR-124-3p is inhibited in SH-SY5Y cells with MPP+ treatment

Firstly, we examined the expression of NEAT1 and miR-124-3p in SH-SY5Y with MPP+ treatment. qRT-PCR uncovered that, after the cells were treated with different concentrations of MPP+, NEAT1 expression level was increased dose-dependently (Figure 1a), whereas miR-124-3p changed oppositely (Figure 1b). Subsequent to 1 mM MPP+ treatment for 12, 24, 48, or 72 h, NEAT1 expression was elevated in SH-SY5Y cells and miR-124-3p expression was declined time-dependently (Figure 1c-d).

**Figure 1.** In SH-SY5Y cells treated with MPP+, NEAT1 expression is up-regulated while miR-124-3p is down-regulated

A, B. SH-SY5Y cells were treated with MPP+ at different concentrations (0, 250, 500, 1000 or 2000 μM), and the expression levels of NEAT1 and miR-124-3p in SH-SY5Y cells were detected by qRT-PCR. C, D. SH-SY5Y cells were treated with 1 mM MPP+ for different times (0, 12, 24, 48, 72 h), and the expression levels of NEAT1 and miR-124-3p were detected by qRT-PCR. All experiments were performed in triplicate. *P < 0.05, ** *P* < 0.01, and *** *P* < 0.001.

### NEAT1 targets miR-124-3p in SH-SY5Y cells

To explore the downstream biological effects after NEAT1 was dysregulated, bioinformatics analysis was performed with StarBase database, and we predicted that there were multiple binding sites on NEAT1 for miR-124-3p. As shown in Figure 2a, there were three putative miR-124-3p binding sites. Next, we constructed luciferase reporter gene vectors containing wild-type sequences of the binding sites (NEAT1-WT) and mutated sequences of the binding sites (NEAT1-MUT-1, NEAT1-MUT-2, NEAT1-MUT-3, NEAT1-MUT-1&2, NEAT1-MUT-1&3, NEAT1-MUT-2&3 and NEAT1-MUT-1&2&3), and subsequently, dual-luciferase report assay was performed. Notably, the luciferase activity of NEAT1-WT was in marked suppression in HEK-293T cells with miR-124-3p mimics transfection, but that of cells co-transfected with NEAT1-MUT-1&2&3 and miR-124-3p mimics was not dramatically changed (Figure 2b). Notably, RIP and RNA pull-down assays further corroborated that, compared with anti-IgG control group, NEAT1 and miR-124-3p were markedly enriched in the immunoprecipitate containing Ago2 (Figure 2c); and miR-124-3p was enriched by biotin-labeled NEAT1, instead of bio-NC (Figure 2d). SH-SY5Y cells were then transfected with NEAT1 overexpression plasmids or siRNAs, and qRT-PCR indicated that NEAT1 depletion could greatly increase miR-124-3p expression in SH-SY5Y cells, while its overexpression could repress miR-124-3p expression (Figure 2e). To sum up, NEAT1 was directly interacted with miR-124-3p, and negatively modulated its expression. Considering the highest knockdown efficiency, si-NEAT1-2 was used for follow-up experiments.

**Figure 2.** NEAT1 targets miR-124-3p in SH-SY5Y cells

A. StarBase database was adopted to predict the recognition sequence of miR-124-3p in NEAT1. B. The luciferase activity of HEK-293 cells co-transfected with NEAT1-WT or NEAT1-Mut and miR-124-3p mimics or NC mimics was examined, to validate the predicted binding site between miR-124-3p and NEAT1. C-D. The interaction between NEAT1 and miR-124-3p in SH-SY5Y cells was verified by RIP and RNA pull-down assays. E. The expression levels of NEAT1 and miR-124-3p in SH-SY5Y cells transfected with pc-NC, si-NC, pc-NEAT1 and si-NEAT1 (si-NEAT1-1, si-NEAT1-2 and si-NEAT1-3) were detected by qRT-PCR. All experiments were performed in triplicate. *P < 0.05, ** *P* < 0.01, and *** *P* < 0.001.

### NEAT1 is a mediator in regulating MPP+-induced inflammation of SH-SY5Y cells via targeting miR-124-3p

To probe the roles of NEAT1 and miR-124-3p in PD, SH-SY5Y cells were divided into four groups after transfection: si-NC group, si-NEAT1 group, si-NEAT1 + NC inhibitor group, and si-NEAT1 + miR-124-3p inhibitors group (Figure 3a). We treated these cells with 1 mM MPP+ for 24 h, and MTT assay showed that MPP+ treatment could raise LDH release, and remarkably repress cell viability; knocking down NEAT1 increased the viability of cells; however, co-transfection of miR-124-3p inhibitors partly eliminated the influence of NEAT1 depletion (Figure 3b-c). Besides, ELISA highlighted that the contents of TNF-α, IL-1β, and IL-6 in MPP+ treated cells were remarkably raised; NEAT1 depletion repressed the inflammatory response of SH-SY5Y cells, and this impact was counteracted by co-transfection of miR-124-3p inhibitors (Figure 3d-f).

**Figure 3.** NEAT1 participates in MPP+-induced injury of SH-SY5Y cells through the regulation of miR-124-3p

SH-SY5Y cells were divided into four groups after transfection: si-NC group, si-NEAT group, si-NEAT + NC inhibitor group, and si-NEAT1 + miR-124-3p inhibitors group. A. The expression of miR-124-3p in SH-SY5Y cells was detected by qRT-PCR after transfection. B. MTT assay was used to detect the viability of SH-SY5Y cells. C. LDH cytotoxicity detection kit was used to determine the injury of SH-SY5Y cells. D-F. The levels of TNF-α, IL-1β, and IL-6 were detected by ELISA. All experiments were performed in triplicate. *P < 0.05, **P < 0.01, and ***P < 0.001.

### NEAT1 can indirectly modulate PDE4B expression via targeting miR-124-3p

Next, we tried to predict and validate the target of miR-124-3p. Through three databases: Starbase, TargetScan, and miRDB, we observed that PDE4B was a downstream candidate target of miR-124-3p (Figure 4a). Following that, dual-luciferase reporter assay was performed, and it indicated that the luciferase activity of cells with PDE4B-WT and miR-124-3p mimics transfection was markedly inhibited, while that of the cells co-transfected with PDE4B-MUT was not significantly repressed (Figure 4b). In addition, qRT-PCR and Western blot indicated NEAT1 depletion suppressed PDE4B expression in SH-SY5Y cells, and that suppression was partially counteracted by co-transfection of miR-124-3p inhibitors (Figure 4c-d), implying that NEAT1 indirectly promoted PDE4B expression via repressing miR-124-3p expression.

**Figure 4.** PDE4B acts as a target of miR-124-3p

A. Bioinformatics was used to predict the binding sites between miR-124-3p and 3ʹ-UTR of PDE4B. B. Dual-luciferase reporter assay verified the targeted binding relationship between miR-124-3p and PDE4B. C-D. After the expression of NEAT1 and miR-124-3p were selectively regulated, qRT-PCR and western blot were used to analyze the expression of PDE4B mRNA and protein. All experiments were performed in triplicate. **P < 0.01, and ***P < 0.001.

### NEAT1 modulates the inflammatory response and injury of SH-SY5Y cells through miR-124-3p/PDE4B/mTOR axis

Next, we tried to figure out the functions of NEAT1/miR-124-3p/PDE4B axis in SH-SY5Y cells. As shown, NEAT1 overexpression repressed miR-124-3p expression in SH-SY5Y cells, and NEAT1 overexpression promoted PDE4B expression, which were counteracted by miR-124-3p mimics co-transfection (Figure 5a-b). Followed by 1 mM MPP+ treatment for 24 h, miR-124-3p overexpression evidently strengthened the viability of neurons, and repressed the release of LDH, and these ameliorative effects were reversed by PDE4B overexpression (Figure 5c-d). What’s more, miR-124-3p overexpression reduced TNF- α, IL-1β, and IL-6 levels, which were offset by PDE4B overexpression (Figure 5e-g). Additionally, miR-124-3p overexpression inhibited the activation of mTOR signaling pathway in SH-SY5Y cells, while PDE4B overexpression counteracted this effect (Figure 5h).

**Figure 5.** NEAT1 regulates the inflammatory response and injury of SH-SY5Y cells through miR-124-3p/PDE4B/mTOR axis

A, B. qRT-PCR and Western blot were used to detect the expression of miR-124-3p and PDE4B in SH-SY5Y cells, respectively, after the cells were transfected with NEAT1 overexpression plasmids, or co-transfected NEAT1 overexpression plasmids and miR-124-3p mimics. SH-SY5Y cells were then divided into four groups: NC mimics group, miR-124-3p mimics group, pc-NC group and pc-PED4B + miR-124-3p mimics group. C. MTT assay was used to detect the viability of SH-SY5Y cells. D. LDH release was determined by LDH cytotoxicity detection kit. E-G. The levels of TNF-α, IL-1β, and IL-6 were detected by ELISA. H. The expression levels of mTOR and p-mTOR protein were detected by Western blot. All experiments were performed in triplicate. **P < 0.01, and ***P < 0.001.

## Discussion

PD, known as a common neurodegenerative disease, features with resting tremor, stiffness, muscle spasm, bradykinesia, and abnormal posture, which seriously reduce people’s life quality [20]. Multiple studies show that dysfunction of dopaminergic neurons and neuroinflammation are the driver of the PD progression [21,22]. Therefore, revealing the mechanism of neuronal apoptosis and neuroinflammatory response is an effective way to find new therapeutic targets for PD. MPP + is a toxic metabolite of MPTP, which can induce most of the pathophysiological changes of PD, and it is widely employed to construct cell model of PD [23]. Therefore, this study adopted MPP + to induce SH-SY5Y to construct PD cell model *in vitro*. In this study, MPP+ treatment induced the cytotoxicity and inflammatory response of SH-SY5Y cells, which is consistent with the previous report [23].

Accumulating studies suggest that lncRNA is associated with the pathogenesis of a variety of diseases, including PD and other neurodegenerative disorders [24–27]. For example, lncRNA-UCA1 is highly expressed in brain tissue of PD mice and SH-SY5Y cells induced by MPP+, which increases neuronal apoptosis and promotes PD progression by increasing α-synuclein expression [28]. LINC-PINT is elevated in the substantia nigra of PD individuals, and its depletion exacerbates the injury of neurons exposed to oxidative stress [29]. In this work, it was demonstrated that NEAT1 was in high expression in SH-SY5Y cells with MPP+ treatment, and its depletion ameliorated the injury of neurons and inflammation response, which is similar with the previous reports [12,30]. Reportedly, lncRNAs can exert its biological functions via multiple mechanism, including functioning as a competitive endogenous RNA to modulate the downstream miRNAs [31,32]. In recent years, reportedly, miRNAs are pivotal regulators in the pathogenesis of neurodegenerative diseases [33–35]. In this work, miR-124-3p expression was decreased in a time- and dose-dependent manner in cells treated with MPP+. As reported, miR-124 modulates the survival, apoptosis, autophagy, mitochondrial function, oxidative stress, and neuroinflammation in PD progression via regulating CDK5, NF-κB, STAT3, Bim, AMPK, Erk and other proteins or pathways [19,36–39]. Reportedly, lncRNA MALAT1 promotes the apoptosis of neurons via repressing miR-124 in PD models [40,41]. Here, NEAT1 was identified to sponge miR-124-3p, and we further verified that, the effects of NEAT1 depletion on neuronal injury and inflammatory response were partly reversed by miR-124-3p inhibitors, implying that the impact of NEAT1 on PD depends on miR-124-3p.

Phosphodiesterase (PDE) is recognized as a vital regulator of various physiological processes. As reported, PDE4 (cAMP-specific) features prominently in the central nervous system, and among the 11 PDE family members. PDE4B, belonging to PDE4, is crucial in regulating neuroinflammation, and PDE4B inhibitors have neuroprotective effects [42–44]. Reportedly, miR-124-3p represses the activity of mTOR signaling by repressing PDE4B expression, and is crucial on neuronal inflammation caused by brain injury [45]. mTOR is a predominant factor of the autophagic process and it is considered as a target to treat neurodegenerative diseases [46]. Our study reported that PDE4B was the direct target of miR-124-3p. Herein, we also authenticated that NEAT1 knockdown could down-regulate PDE4B expression via promoting miR-124-3p expression in SH-SY5Y cells. Additionally, overexpressing miR-124-3p repressed the inflammatory response and injury of SH-SY5Y cells induced by MPP+ via suppressing PDE4B. Notably, overexpressing miR-124 significantly repressed the phosphorylation level of mTOR. These results suggested that NEAT1 could probably activate mTOR signaling through regulating miR-124-3p/PDE4B axis in neurons during PD pathogenesis, to aggravate the neuroinflammation and neuron death.

## Conclusion

To recapitulate briefly, NEAT1 is up-regulated and miR-124-3p expression is reduced in SH-SY5Y cells with MPP+ inducement. Functionally and mechanistically, NEAT1 aggravates the injury of SH-SY5Y cells via regulating miR-124-3p/PDE4B axis. We clarify the molecular regulatory mechanism of NEAT1 in the pathogenesis of PD, proving that NEAT1/miR-124-3p/PDE4B axis is involved in the progression of PD (Figure 6). Animal models, in the future, are needed to further validate our conclusion.

**Figure 6.** Graphic Abstract. NEAT1 functions as a molecular sponge to regulate miR-124-3p, PDE4B and mTOR signaling, to mediate the neurological inflammation and injury in PD

## Highlights

1. NEAT1 expression is up-regulated in SH-SY5Y cells treated with MPP+.

2. NEAT1 regulates neuron’s viability and apoptosis via miR-124-3p/PDE4B axis.

3. NEAT1 may be a promising therapy target for PD.
